RETRACTED

# Correlation between NLR, PLR, and LMR and Disease Activity, Efficacy Assessment in Rheumatoid Arthritis

**DOI:** 10.1155/2021/4433141

**Published:** 2021-10-22

**Authors:** Mei Li, Lihu Xie

**Affiliations:** The First Affiliated Hospital, Department of Rheumatology and Immunology, Hengyang Medical College, University of South China, Hengyang, Hunan 421001, China

## Abstract

**Objective:**

To analyze the value of neutrophil-lymphocyte ratio (NLR), platelet-lymphocyte ratio (PLR), and lymphocyte-monocyte ratio (LMR) in the evaluation of disease activity and efficacy in patients with rheumatoid arthritis (RA).

**Methods:**

The clinical data of 132 newly diagnosed RA patients admitted to our hospital from November 2018 to January 2020 were retrospectively analyzed, and the NLR, PLR, and LMR were calculated. According to the 28-joint disease activity score (DAS28), all patients was divided into the remission group (*n* = 40) and the active group (*n* = 92). According to the curative effect of the active group, the patients were divided into the effective group (*n* = 61) and the ineffective group (*n* = 39). Logistic regression analysis of clinical data was to determine the influencing factors of RA disease activity. The receiver operating characteristic curve (ROC) was used to evaluate the predictive value of NLR, PLR, and LMR on disease activity and efficacy of RA.

**Results:**

The number of cases of smoking history, the number of cases of drinking history, and NLR, PLR, CRP, and ESR levels of patients in the active group were higher than those of the remission group, and the LMR level was lower than that of the remission group; the differences were statistically significant (*P* < 0.05). The results of multivariate logistic regression analysis showed that NLR, PLR, LMR, CRP, and ESR were independent influencing factors of disease activity in RA patients (*P* < 0.05). The AUC of NLR, PLR, and LMR on the disease activity of RA patients was 0.872, 0.821, and 0.824, the sensitivity was 87.6%, 70.2%, and 69.3%, and the specificity was 75.6%, 76.8%, and 84.3%, respectively. The NLR and PLR values of the effective group were lower than those of the ineffective group, and the LMR values were higher than those of the ineffective group, and the differences were statistically significant (*P* < 0.05). The AUC of NLR, PLR, and LMR on the efficacy of RA patients was 0.756, 0.732, and 0.779, the sensitivity was 68.4%, 60.2%, and 67.9%, and the specificity was 83.2%, 86.4%, and 85.1%, respectively.

**Conclusion:**

NLR, PLR, and LMR are the independent factors that affect the disease activity of RA patients and can better evaluate the disease activity and efficacy of RA.

RETRACTED

## 1. Introduction

Rheumatoid arthritis (RA) is a chronic autoimmune disease with unknown etiology. Its clinical symptoms are mainly manifested by joint injuries such as hands and feet, which are difficult to reverse. As the disease progresses, it may lead to joint malformation or even loss of function, resulting in difficulty for patients to take care of themselves [1]. At present, the treatment of RA is mainly to relieve the clinical symptoms and control the disease progression. However, the long-term clinical remission rate is still relatively low. Therefore, how to better evaluate the disease status of patients with early RA and develop appropriate treatment plans to achieve better efficacy has always been one of the focuses of clinicians. It is known that inflammation is closely related to the occurrence and development of RA, and C-reactive protein (CRP) and erythrocyte sedimentation rate (ESR) are commonly used as inflammatory indicators to evaluate RA. ESR and CRP can predict the severity of RA, but they are difficult to predict the therapeutic effect. At the same time, their measurement is complex and their clinical application is limited [2, 3]. Peripheral blood cell count ratio is a relatively new inflammatory indicator, including neutrophil-lymphocyte ratio (NLR), platelet-lymphocyte ratio (PLR), and lymphocyte-monocyte ratio (LMR). These indicators can better reflect the systemic inflammation and are easy to obtain and low in cost. They have been used for the evaluation of the degree of inflammation and the prognosis of curative effects in rheumatism, tumor, cardiovascular disease, and respiratory system disease [4–6]. However, there are still few studies on whether NLR, PLR, and LMR can be used to judge the disease activity and treatment effect of RA patients. Therefore, this study retrospectively analyzed the clinical data of newly diagnosed RA patients in our hospital and explored the value of NLR, PLR, and LMR in disease activity and efficacy evaluation, and the details are given as follows.

## 2. Materials and Methods

### 2.1. Research Object

The clinical data of 132 newly diagnosed RA patients admitted to our hospital from November 2018 to January 2020 were retrospectively analyzed. There were 27 males and 105 females, aged from 30 to 70 years, with an average age of (50.06 ± 10.65) years. Inclusion criteria: meet the diagnostic criteria of RA in “2015 American College of Rheumatology Guideline for the Treatment of Rheumatoid Arthritis” [7], no RA-related treatment, and complete case data. Exclusion criteria: severe organ dysfunction such as the heart, liver, and kidney, associated with other immune system diseases, severe diseases of the blood system, and combined with malignant tumor. According to 28-joint disease activity score 28 (DAS28), patients were divided into the remission group (*n* = 40) and the activity group (*n* = 92). After standard treatment, according to clinical efficacy, the active group was divided into the effective group (*n* = 61) and the ineffective group (*n* = 39). All information obtained was agreed by the subjects and informed consent was signed. This study has been approved by the ethics committee of our hospital.

RETRACTED

### 2.2. Research Methods

#### 2.2.1. Clinical Data Collection

Gender, age, underlying diseases, education level, DAS28 score, and other general information of all patients were recorded. DAS28 ≤ 2.6 was regarded as remission. DAS28 > 2.6 points are regarded as disease activities. Fasting venous blood of all subjects was collected in the morning, and blood routine tests were performed by an automatic blood analyzer (XT-2000I, XISen Micron, Japan) (reference value: neutrophils 2.0–7.5×109/L, lymphocytes 0.8–4.0×109/L, platelets 100–300×109/L, and monocytes 0.3–0.8×109/L), and calculate NLR, PLR, and LMR. CRP (reference value: 5–10 mg/L) and ESR (reference value: 0–20 mm/h) were detected.

#### 2.2.2. Efficacy Evaluation

Patients in the activity group were evaluated after 3 months of standard treatment. Effective: clinical symptoms improved or disappeared, joint function improved, CRP and other indicators improved ≥50%, and patients can take care of themselves or basic self-care. Invalid: no remission or even aggravation of clinical symptoms, the improvement of CRP and other indicators<50%, and patients still have difficulty in self-care.

### 2.3. Statistical Methods

SPSS 22.0 software was used for processing. The measurement data were expressed as mean ± standard deviation (mean ± SD), and the counting data were expressed as (%). Analysis of variance was used for multigroup comparison of measurement data between groups, and the *t*-test was used for pial comparison. Statistical data were tested by the *χ*^2^ test. The factors of disease activity were analyzed by binary multifactor logistic regression. Receiver operating characteristic curve (ROC) and area under curve (AUC) were used to evaluate the prediction of NLR, PLR, and LMR for disease activity and efficacy. *P* < 0.05 was considered statistically significant.

## 3. Results

### 3.1. Comparison of Clinical Data between the Remission Group and Activity Group

The number of smoking patients and drinking patients, NLR, PLR, CRP, and ESR levels in the activity group were higher than those in the remission group, while LMR levels were lower than those in the remission group, and the differences were statistically significant (*P* < 0.05), as given in Table 1.

RETRACTED

### 3.2. Multivariate Logistic Regression Analysis of Disease Activity in RA Patients

Multivariate logistic regression analysis showed that NLR, PLR, LMR, CRP, and ESR were independent influencing factors of RA patients (*P* < 0.05), as given in Tables 2 and 3.

### 3.3. Predictive Value of NLR, PLR, and LMR for Disease Activity and Remission in RA Patients

The AUC of NLR for differential diagnosis of disease activity and remission in RA patients was 0.872 (95% CI: 0.769–0.918). When the optimal cutoff value was 0.659, the sensitivity and specificity were 87.6% and 75.6%, respectively. The AUC of PLR for the differential diagnosis of disease activity and remission in RA patients was 0.821 (95% CI: 0.749–0.889). When the optimal cutoff value was 0.493, the sensitivity and specificity were 70.2% and 76.8%, respectively. The AUC of LMR for differential diagnosis of disease activity and remission in RA patients was 0.824 (95% CI: 0.749–0.896). When the optimal cutoff value was 0.555, the sensitivity and specificity were 69.9% and 84.3%, respectively, as given in Table 4 and Figure 1.

### 3.4. Comparison of NLR, PLR, and LMR among Patients with Different Therapeutic Effects

According to the efficacy evaluation criteria, 61 patients were effective and 39 patients were ineffective after treatment. Before or after treatment, NLR and PLR values in the effective group were lower than those in the ineffective group, while LMR values were higher than those in the ineffective group, and the differences were statistically significant (*P* < 0.05), as given in Table 5.

### 3.5. Predictive Value of NLR, PLR, and LMR for the Efficacy of RA Patients

The AUC of NLR for RA patients was 0.756 (95% CI: 0.672–0.899). When the optimal cutoff value was 0.543, the sensitivity and specificity were 68.4% and 83.2%, respectively. The AUC of PLR for RA patients was 0.732 (95% CI: 0.665–0.897). When the optimal cutoff value was 0.468, the sensitivity and specificity were 60.2% and 86.4%, respectively. The AUC of LMR for RA patients was 0.779 (95% CI: 0.682–0.911), when the optimal cutoff value was 0.553, the sensitivity and specificity were 67.9% and 85.1%, as given in Table 6 and Figure 2.

## 4. Discussion

The etiology of RA is complex, involving many factors such as heredity, infection, and sex hormones. RA is mainly associated with inflammatory changes in joints. In its early stage, RA mainly involves peripheral joints and may lead to the formation of pannus and synovitis. With disease progression, disease can get involved cartilage and bone, osteoporosis, and patients can appear because of the function of the joints, structural damage of joint deformity, loss of ability to care for life, and some patients even in extraarticular manifestations or involving the cardiovascular, respiratory, kidney, nerve, and multiple systems all over the body [8–10]. There is currently no complete cure for RA. The treatment of RA is long-term, and the main purpose is to control the progress of inflammation, relieve joint injury, and improve the self-care ability of patients. However, the long-term remission rate of RA patients is still relatively low so far, so it is very important to effectively monitor the patient's condition in the long-term treatment.CRP, ESR, DAS28, and other indicators can be used for the evaluation of RA disease activity and efficacy. However, CRP and ESR were also susceptible to a variety of factors not related to inflammation, such as age, gender, anemia, and therapeutic drugs, and were more complex to detect than peripheral blood counts. Therefore, all the above indicators have their limitations, and it is of great significance to find other simple and feasible clinical markers for the long-term management of RA patients. At present, the ratio of NLR, PLR, LMR, and other peripheral blood counts to evaluate systemic inflammation has been widely applied in clinical practice. For example, the increase of NLR and PLR often indicates poor prognosis of tumor; besides, in patients with ulcerative colitis, it is positively correlated with disease activity, but the LMR level is negatively correlated [11, 12]. The results of this study showed that NLR, PLR, LMR, CRP, and ESR were all independent influencing factors of RA patients' disease activity. The reason was that inflammatory cytokines were closely related to the occurrence and development of various inflammatory diseases, which may aggravate the synovial inflammatory response and promote pannus formation in RA patients. In addition, neutrophils, platelets, monocytes, and other peripheral blood cells are involved in the production of such inflammatory cytokines and can secrete a large number of free oxygen free radicals and lyase to assist in the effect, so the fluctuation of the above indicators can have an important impact on the activity of RA [13, 14]. NLR, PLR, and LMR have a good value for judging RA disease activity, with AUC values of 0.872, 0.821, and 0.824, respectively, indicating that NLR, PLR, and LMR are the same as CRP and ESR and can be used as important indicators in assessing RA disease activity. However, compared with CRP and ESR, NLR, PLR, and LMR are enumeration ratios, which are not only simple to operate but also can eliminate the effects of physiological and physical factors on the value of leukocyte subtypes as much as possible, reflect the degree of inflammation more objectively, and remain relatively stable. Due to their special pathogenesis, the serum levels of inflammatory factors such as tumor necrosis factor-*α* in patients with RA are significantly higher than those in the normal population. When RA is in the active stage, such factors can promote the differentiation and survival of neutrophils and their migration to synovium by increasing the secretion of the granulocyte colony-stimulating factor. At the same time, a large number of reactive oxygen species and enzymes that damage joint tissues are released, which is one of the important mechanisms by which the peripheral blood count cells can be used to judge the disease activity of RA [15, 16]. Studies showed that platelets may play a role in aggravating and maintaining inflammation in the pathogenesis of RA [17]. It is difficult to detect the increase of platelets in the joints of RA patients at rest, while a large number of platelet-specific proteins can be detected in the joint synovial fluid and serum of RA patients at the active stage. In addition, during disease activity, more T cells will accumulate in the synovial membrane, resulting in a decrease in the number of T cells in the peripheral circulation, resulting in a lower lymphocyte detection count [18, 19]. Therefore, patients with RA in the active stage may present with various manifestations such as neutrophil, platelet elevation, and lymphocyte decline, which makes the ratio of peripheral blood cell count significantly different from that in the remission stage.The results of this study also showed that no matter before or after treatment, NLR, PLR, and LMR values were significantly different between the effective group and the ineffective group. NLR, PLR, and LMR values have a good value in the prediction of efficacy, which can be used as an important basis for the treatment plan of patients. Therefore, for RA patients with poor predictive efficacy in clinical treatment, more measures can be taken in combination with disease control to avoid delaying early treatment due to ineffective conventional treatment.

RETRACTED

## 5. Conclusion

NLR, PLR, and LMR are independent influencing factors of disease activities of RA and have a good value for evaluating disease activities and efficacy. Due to their effectiveness and simplicity, they can be used as reference indicators for long-term clinical monitoring of RA.

## Figures and Tables

**Figure 1:** Predictive value of NLR, PLR, and LMR for disease activity in RA patients. The closer to the upper left of the standard line, the higher the forecast value of the indicator. If it is located at the lower right of the standard line, there is no forecast value.

**Figure 2:** Predictive value of NLR, PLR, and LMR for efficacy in RA patients. The closer to the upper left of the standard line, the higher the forecast value of the indicator. If it is located at the lower right of the standard line, there is no forecast value.

**Table 1:** Comparison of clinical data between the remission group and activity group (*n*, %, mean ± SD).

Variable	Remission group (*n* = 40)	Activity group (*n* = 92)	*t/χ* ^2^	*P*
Male/female	10/30	17/75	0.177	0.821
Age	48.52 ± 9.36	52.72 ± 11.35	2.396	0.039
Smoking	6 (15.00)	33 (35.87)	4.469	0.029
Drinking	10 (25.00)	42 (45.65)	4.233	0.031
Hypertension	9 (22.50)	22 (23.91)	0.296	0.997
Diabetes	4 (10.00)	15 (16.30)	0.532	0.698
NLR	2.37 ± 0.96	3.61 ± 1.09	4.022	<0.001
PLR	149.86 ± 39.57	195.33 ± 46.82	4.631	<0.001
LMR	4.71 ± 1.88	3.94 ± 1.69	3.851	<0.001
CRP (mg/L)	13.88 ± 8.65	26.71 ± 9.58	8.005	<0.001
ESR (mm/h)	22.36 ± 12.57	46.31 ± 32.89	5.644	<0.001

**Table 2:** Assignment value of multivariate logistic regression analysis.

Variable	Assignment value
Smoking	“No” = “0”; “yes” = “1”
Drinking	“No” = “0”; “yes” = “1”

**Table 3:** Multivariate logistic regression analysis of disease activity in RA patients.

Variable	B	Wald	OR	95% CI	*P*
Smoking	0.283	5.223	1.309	0.623–2.641	0.196
Drinking	0.226	3.257	1.255	0.689–1.859	0.372
NLR	0.196	9.361	1.231	1.339–2.465	0.013
PLR	0.257	6.333	1.284	1.127–1.893	0.028
LMR	−0.343	3.284	0.723	0.496–0.975	0.011
CRP	0.179	5.643	1.212	1.439–1.996	0.016
ESR	0.366	7.532	1.489	1.123–2.997	0.027

**Table 4:** Predictive value of NLR, PLR, and LMR for disease activity in RA patients.

Index	AUC	Asymptotically approaching 95% confidence interval		Optimum truncation value	Sensitivity (%)	Specific degrees (%)
		The lower limit	Ceiling			
NLR	0.872	0.769	0.918	0.659	87.6	75.6
PLR	0.821	0.749	0.889	0.493	70.2	76.8
LMR	0.824	0.749	0.896	0.555	69.9	84.3

**Table 5:** The level of NLR, PLR, and LMR between patients with different curative effects (*n*, mean ± SD).

Variable		Effective group (*n* = 61)	Invalid group (*n* = 39)	*t*	*P*
NLR	Before	3.16 ± 1.33	4.23 ± 1.25	4.278	<0.001
	After	2.23 ± 1.21	3.35 ± 1.09	3.968	<0.001
PLR	Before	186.54 ± 41.33	227.69 ± 46.85	4.221	<0.001
	After	144.96 ± 45.31	196.57 ± 51.33	4.621	<0.001
LMR	Before	4.32 ± 1.76	3.29 ± 1.41	3.953	<0.001
	After	4.63 ± 1.29	3.59 ± 1.33	3.889	<0.001

**Table 6:** Predictive value of NLR, PLR, and LMR for the efficacy of RA patients.

Index	AUC	Asymptotically approaching 95% confidence interval		Optimum truncation value	Sensitivity (%)	Specific degrees (%)
		The lower limit	Ceiling			
NLR	0.7756	0.672	0.899	0.543	68.4	83.2
PLR	0.732	0.665	0.897	0.468	60.2	86.4
LMR	0.779	0.682	0.911	0.553	67.9	85.1

RETRACTED

## Data Availability

The data used to support the findings of this study are available from the corresponding authorupon request.
